# College Students' Mental Health Support Based on Fuzzy Clustering Algorithm

**DOI:** 10.1155/2022/5374111

**Published:** 2022-08-16

**Authors:** Zengliu Xu

**Affiliations:** China Academy of Art, Hangzhou, Zhejiang 310002, China

## Abstract

There are some problems in the active participation of college students in ideological and mental health support services in China, such as low attention, low participation, and high data redundancy. Based on this, this paper studies the active participation of college students' ideological and mental health support service based on fuzzy cluster analysis algorithm. Compared with the disadvantages of the current mainstream discrete optimization analysis models on mental health (such as high-dimensional enterprise model, Dajiaweikang model, and short-range group control model), which need to set the known data gradient interval, this paper creatively adopts the fuzzy cluster analysis algorithm, based on the characteristics of different types of college students' ideological and mental health problems. Combined with the improved star discrete analysis model, this paper constructs the active participatory evaluation strategy of college students' ideological and mental health support services. On this basis, the model can not only record and store the participatory data of ideological and mental health support for students of different grades but also match and track different types of data based on special framework conditions, so as to achieve numerical normal analysis and directional matching for the data coupling mode of college students' ideological and mental health support services. On the other hand, the Planck constant factor is used to classify different types of ideological and psychological factor data, and combined with the idea of fuzzy clustering, the hierarchical analysis and quantitative calibration of different types of data groups are realized, so as to improve the reliability and authenticity of the active participation in college students' mental health support services. The results show that this star discrete analysis model can analyze the active participation of college students' ideological and mental health support services according to the data matching degree of different levels and can effectively improve the analysis efficiency of data vectors. Compared with the traditional research methods on the active participation of college students' ideological and mental health support services, this method can realize the matching and tracking of different types of data, so as to make a numerical and normal analysis on the data coupling mode of college students' ideological and mental health support services.

## 1. Introduction

At present, college students in different regions have great differences in mental health, which is mainly reflected in the psychological change process in the process of daily life and learning [1]. As colleges and universities have the characteristics of multiregional cultural collection, college students come from all over the country and live in different environments since childhood. However, students who grow up in different cultures and social customs tend to show different ways of thinking, value orientation, interpersonal communication, and other aspects. College students are used to thinking from the cultural model of their own region and measuring local college students or college students from other regions with their own regional values and behaviors, so as to deepen their prejudice against other regional cultures in life and interpersonal communication. In recent years, with the development of big data, intelligent algorithms, and various data analysis methods and technologies, many experts and scholars have gradually adopted the method of “intelligent data analysis method + mental health diagnosis” in the study of mental health problems [2]. On the other hand, school students also conduct self-diagnosis and enlightenment according to different types of mental health problems, mainly including mutual chat, emotional catharsis, and book learning [3]. In terms of mental health support services for college students, most colleges and universities have carried out customized mental health support service consulting rooms [4]. For example, most colleges and universities regularly carry out different levels of mental health curriculum education and mental health questionnaire survey activities for students, which can effectively improve students' mental health satisfaction to a certain extent, but there are still deficiencies in the intelligent classification and customized high-efficiency matching of mental health support services [5]. Based on this background, this paper studies the active participation survey satisfaction of college students' ideological and mental health support service and puts forward the application and reliability analysis model of college students' ideological and mental health service based on fuzzy cluster analysis algorithm.

At present, although most colleges and universities have established the curriculum system of mental health education, some colleges and universities still have outdated educational ideas and backward ideas, which leads to the lack of understanding of mental health education in colleges and universities, which greatly reduces the implementation effect of mental health education among college students. Although most colleges and universities have established the curriculum system of mental health education, some colleges and universities still have outdated educational ideas and backward ideas, which leads to the lack of understanding of mental health education in colleges and universities, which greatly reduces the implementation effect of mental health education among college students. In view of the problems of high laziness, insufficient attention, and high data redundancy in the existing ideological and mental health support services for college students, this paper studies the application of star discrete data analysis model based on fuzzy cluster analysis algorithm in the optimization of support service structure in college students' ideological and mental health, which is mainly divided into four parts. Section 1 introduces the research background, research structure, and innovation of college students' ideological and mental health. Section 2 introduces the research status of the evaluation methods of college students' ideological and mental health support service enthusiasm and the analysis of college students' ideological and mental health data in different regions at home and abroad. Section 3 constructs the evaluation method of college students' ideological and mental health support service based on star discrete analysis model based on fuzzy cluster analysis algorithm and constructs the discrete database of college students' ideological and mental health information by using Planck constant curvature coupling analysis equation method. Section 4 tests the reliability of star discrete analysis model based on fuzzy cluster analysis algorithm in the evaluation method of college students' ideological and mental health support service enthusiasm and draws a conclusion through the coupling analysis of the experimental data.

Compared with the disadvantages of the current mainstream discrete optimization analysis models on mental health (such as high-dimensional enterprise model, Dajiaweikang model, and short-range group control model), which need to set the known data gradient interval, the innovation of this paper is that, through the fuzzy cluster analysis algorithm, according to the characteristics of different types of college students' ideological and mental health problems, combined with the improved star discrete analysis model, this paper constructs the active participatory evaluation strategy of college students' ideological and mental health support services. On this basis, the model can not only record and store the participatory data of ideological and mental health support for students of different grades, but also realize the matching and tracking of different types of data based on the special framework conditions, so as to realize the numerical and normal operation of the data coupling mode of college students' ideological and mental health support services. On the other hand, Planck constant factor is used to classify different types of ideological and psychological factor data, and fuzzy clustering method is used to carry out hierarchical analysis and quantitative calibration for different types of data groups, so as to improve the overall reliability and authenticity.

## 2. Related Work

At this stage, most of the research on college students' mental and ideological health focuses on the value and stability of mental and ideological health, and little research with intelligent characteristics is carried out in the support customized service of characteristic mental health [6]. Aiming at the uncontrollable factors of college students' active participation in mental health support services, Lee and other scholars used the three-dimensional high-intensity fingertip algorithm to analyze the impact of different types of data groups and high-intensity matching tracking strategies and found that different types of mental health services have differences. High-intensity matching of different data can be realized through this strategy [7]. Tian and other scholars put forward a high-intensity integration model combined with the cultural characteristics of local colleges and universities to solve the problem of insufficient trust of college students in the process of mental health diagnosis [8]. In order to solve the problem of transition analysis of college students' enthusiasm for support services, Duan and other scholars proposed a continuous matching blending model based on flexible strategies of high-value analysis with different intensities, so as to adopt more targeted high-value data analysis for different types of college students' mental health thoughts [9]. Caldas and other scholars put forward a stability sum analysis method based on high driving strategy according to the stability difference factors of college students in ideological health. Through confirmatory experiments, it is found that this strategy has good value tracking effect [10]. After investigating 1000 college students, Gavioli and other scholars found that most male students had mental health problems, and their internal correlation was disturbed to varying degrees. Therefore, they proposed a research platform for college students' mental health support based on Turing analysis algorithm [11]. According to different types of college students, Pramod and other scholars adopt layered strategies to realize the customized cultivation of college students' ideological and mental health and put forward a highly targeted mental health counseling strategy, but it needs the cooperation of college students [12]. Moazzen and other scholars classify and analyze the mental health support services of college students with different attributes, realize the differentiated management of college students' mental health problems, and then realize the matching analysis of their internal relevance. The experimental results show that this method has strong stability and customized analysis effect [13]. Qiao and other scholars used different levels of iterative stacking analysis to realize the normalized analysis of different degrees of mental health problems and proposed a hybrid stacking service strategy based on high-intensity memory analysis [14]. Tsang and other scholars rely on different types of databases to realize customized mental health services for college students of different grades and conduct one-to-one reinforcement analysis according to the participation of college students [15].

Domestic and foreign researches on blustering Based on different types of mental analysis methods are rarely carried out [16–18]. Cluster analysis groups and classifies the seemingly disordered objects (such as tables, people, trees, emotions, and ideas) and classifies them according to the characteristics of individuals or samples, so that individuals in the same category have as high homogeneity as possible, while different categories have as high heterogeneity as possible, so as to better understand the research objects. Birds of a feather flock together. With the help of clustering analysis algorithm, it can help us spy on the data differences between different populations. Therefore, this method is also applied to the practice of user classification based on quantitative data. On the other hand, in the research link of active participation in support services, there is also a lack of matching value analysis mode involving the combination of different types of data classification strategies and fuzzy evaluation strategies, which leads to different degrees of deviation in the process of matching analysis [19–21]. Therefore, it is of great significance to study the intelligent analysis strategy and application of the active participation of college students' mental health support services based on fuzzy clustering [22].

## 3. Methodology

### 3.1. Application of Star Discrete Analysis Model Based on Fuzzy Clustering in Support Service Structure Optimization

In engineering technology and economic management, it is often necessary to classify some indicators according to certain standards (similar degree or affinity, etc.). For example, classify organisms according to some properties, classify air quality according to the properties of air, classify product quality in industry, classify project scale in engineering, classify graphics in image recognition, classify soil in geology, and classify water quality in water resources. These mathematical methods of classifying objective things according to certain standards are called cluster analysis, which is a classification method of “clustering things” in multivariate statistics. However, in science, technology, and economic management, there is no clear division between classes of many things, the boundary is fuzzy, and the relationship between them is fuzzier. For the classification of this kind of things, fuzzy mathematics method is generally used. We call the clustering analysis using fuzzy mathematics method as fuzzy clustering analysis. Fuzzy clustering analysis algorithm is one of the common strategies for high-intensity characterization analysis of massive data. This method realizes the multidimensional two-in-one classification of its internal data by adopting the coupling analysis idea of clustering center, using different types of high-intensity data analysis methods and combining its internal correlation characteristics. The strategy often used in this method is to divide the predata into multiple levels according to its discrete type and correlation law. When it is divided into multiple level data groups, its internal matching and flexible disturbance characteristics can be analyzed according to its internal high-intensity data flow and then calculate the distance of different types of data centers, the vector representation and regularity matching of the data group are realized, and the iterative operation and efficient classification of degrees of freedom of the data group are realized by using filtering rules [23]. This process needs to be carried out in a cycle until the optimal data matching criteria are met. The data analysis process of star discrete analysis model based on fuzzy clustering in supporting service structure optimization is shown in Figure 1. The economic meaning of star model is that all changes in the economic aggregate are mainly caused by the changes of individuals with different behaviors, and not all individuals react to an economic signal at the same time and interact with each other. Unlike discrete transfer models, the transfer of smooth transfer regression models is a continuous process based on transferred variables (Hansen, 1999). When the time of district system transformation is uncertain and the new district system has not yet been produced, the smooth transfer regression model effectively reflects the district system transfer behavior, so the model can capture the dynamic characteristics of variables in the transfer stage. At the same time, it has the characteristics of nonlinearity and zoning transfer, which makes the model an important tool to study economic variables. Fuzzy clustering analysis algorithm is one of the common strategies for high-intensity characterization analysis of massive data. This method realizes the multidimensional two-in-one classification of its internal data by adopting the coupling analysis idea of clustering center, using different types of high-intensity data analysis methods and combining its internal correlation characteristics [24]. The strategy often used in this method is to divide the predata into multiple levels according to its discrete type and correlation law. When it is divided into multiple level data groups, its internal matching and flexible disturbance characteristics can be analyzed according to its internal high-intensity data flow, and then calculate the distance of different types of data centers. The vector representation and regularity matching of the data group are realized, and the iterative operation and efficient classification of degrees of freedom of the data group are realized by using filtering rules [25]. This process needs to be carried out in a cycle until the optimal data matching criteria are met, and the data analysis process of star discrete analysis model based on fuzzy clustering in supporting service structure optimization is shown in Figure 1.

### 3.2. The Analysis Process of Star Discrete Analysis Model in the Active Participation of Support Services

After establishing the star discrete analysis model based on fuzzy cluster analysis algorithm, it is necessary to quantify and rank the analysis process of its active participation in college students' ideological and mental health support services. Therefore, the first step is to design the norm value, expectation value, and dispersion value of star discrete analysis model based on fuzzy cluster analysis algorithm. The normal value function *R*(*x*), the expected value function *Y*(*x*), and the dispersion value function *T*(*x*) used in this study are

(1) $$\begin{array}{c} R\left(x\right)=\sqrt{\sum_{k=1}^{p}\frac{x_{k}^{2}+x_{k-1}^{2}}{x_{k+1}^{2}}+\frac{\sum_{k=1}^{p}x_{k}^{2}/x_{k+1}^{2}}{k{\bar{x}}_{p}}},\\ Y\left(x\right)=\frac{p!}{1+{\bar{x}}_{p+k-1}}\sqrt{\frac{x_{1}+x_{k}+x_{p}}{{\bar{x}}_{p+k-1}}},\\ T\left(x\right)=\frac{\sqrt{1+\sum_{k=1}^{p}{\left(x_{k}+{\bar{x}}_{p}\right)}^{2}}}{k+{\bar{x}}_{p}}. \end{array}$$

*x*_*k*_ is the data of college students' ideological and mental health, *p* is the data of active participation in support services, *k* is the type of mental health support, and ${\bar{x}}_{p}$ is the standard mean value of college students' ideological and mental health.

After the normal value function and expected value function are processed by fuzzy cluster analysis, the corresponding expression is

(2) $$\begin{array}{c} R^{\prime }\left(x\right)=\sqrt{1+\frac{\sqrt{1+\sum_{k=1}^{p}x_{k}^{2}/x_{k+1}^{2}}}{k+\sum_{k=1}^{p}{\left(x+{\bar{x}}_{p}/1+{\bar{x}}_{p}\right)}^{2}}},\\ Y^{\prime }\left(x\right)=\frac{\left(p+1\right)!/p{\bar{x}}_{p+k-1}+\sqrt{x_{1}+x_{k}+x_{p}/{\bar{x}}_{p+k-1}}}{x_{k}+x_{p}},\\ T^{\prime }\left(x\right)=\frac{1+\sqrt{100p+\sum_{k=1}^{p}{\left(x_{k}+{\bar{x}}_{p}\right)}^{2}/k+p\sum_{k=1}^{p}{\left(x+{\bar{x}}_{p}/1+{\bar{x}}_{p}\right)}^{2}}}{1+{\bar{x}}_{p}}. \end{array}$$

*x*_*k*_ is the data of college students' ideological and mental health, *p* is the data of active participation in support services, *k* is the type of mental health support, and ${\bar{x}}_{p}$ is the standard mean value of college students' ideological and mental health. Input different types of mental health data sets into this star discrete analysis model. The simulation analysis results of its active participation in support services in quantitative evaluation are shown in Figure 2.

It can be seen from Figure 2 that, after fuzzy cluster analysis, the matching degree of internal relevance data group and active participation of support services of different types of data groups varies greatly, which is mainly presented in different types of high-intensity analysis, and after two-dimensional analysis of different types of data groups, their internal relevance presents different change trends. This is because different types of college students' mental and ideological health have different value matching analysis strategies, and their corresponding data group types also have different analysis results. The vector modulus function *F*(*x*), high-value degree analysis function *G*(*x*), and low strength error function involved in this stage are *H*(*x*):

(3) $$\begin{array}{c} F\left(x\right)=1+\frac{k}{m\left|x\right|}\sqrt{{\left|x\right|}^{2}+m\left|x\right|+\sqrt{\left|x\right|}/k\left|x\right|+m{\left|x\right|}^{2}+k},\\ G\left(x\right)=\frac{\sqrt{1+m\left|x\right|/k+1\sum_{k=1}^{m}\sqrt{m{\left|x\right|}^{2}+m\left|x\right|+\sqrt{\left|x\right|}}/m\left|x\right|+k{\left|x\right|}^{2}+mk}}{m\left|x\right|+k\sqrt{\left|x\right|}},\\ H\left(x\right)=\frac{\sqrt{\left(1-G\left(x\right)/km\right)}+\sqrt{kF^{2}\left(x\right)+mF\left(x\right)/kF\left(x\right)+mx}}{m+k}. \end{array}$$

|*x*| is the module length of college students' mental and ideological health data vector and *m* and *k* are the number and type of support service active participation data groups, respectively. After fuzzifying the above three functions, the corresponding expression is

(4) $$\begin{array}{c} F^{\prime }\left(x\right)=m\sqrt{1+\frac{k}{m\left|x\right|}\sqrt{\frac{{\left|x\right|}^{2}+m\left|x\right|+\sqrt{\left|x\right|}}{k\left|x\right|+m{\left|x\right|}^{2}+k}}},\\ G^{\prime }\left(x\right)=\frac{k\sqrt{m+\sum_{k=1}^{m}\sqrt{m{\left|x\right|}^{2}+m\left|x\right|+\sqrt{\left|x\right|}}/m\left|x\right|+k{\left|x\right|}^{2}+mk+k-1/m\left|x\right|+k{\left|x\right|}^{2}+mk}}{mk+m+k},\\ H^{\prime }\left(x\right)=\frac{\sqrt{\sum_{k=1}^{m}\left(1-G\left(x\right)/km\right)+kF^{2}\left(x\right)+mF\left(x\right)/kF\left(x\right)+mx/mF\left(x\right)+kx}}{\sqrt{mk+mkF^{2}\left(x\right)+\left(m+1\right)F\left(x\right)/kF\left(x\right)+mkx}}. \end{array}$$

|*x*| is the module length of college students' mental and ideological health data vector and *m* and *k* are the number and type of support service active participation data groups, respectively.

The second step is to determine the strength function value of star discrete analysis model for the analysis of college students' mental health data. This process requires the introduction of participatory value evaluation function *Q*(*x*) and stable value function *W*(*x*) based on fuzzy cluster analysis strategy. Their mathematical expressions are as follows:

(5) $$\begin{array}{c} Q\left(x\right)=1+\sqrt{\frac{1+\sum_{j=1}^{p}\left(jx_{j}^{2}+{\bar{x}}^{3}\right)}{2+\sum_{k=1}^{p}{\left(kx_{k}^{2}-{\bar{x}}^{2}\right)}^{2}}},\\ W\left(x\right)=1-\sqrt{\frac{kp+\sum_{k=1}^{p}{\left(kx_{k}^{2}-{\bar{x}}^{2}\right)}^{2}}{p\bar{x}}}. \end{array}$$

*x* represents different sample groups of college students' mental health data, *k* and *j* represent different numbers, and *p* represents the corresponding limit numbers in different groups. The function set determined by the central data used in the subsequent simulation experiment is as follows:

(6) $$\begin{array}{c} F\left(x\right)=\frac{\left(l+r\right)\left(\sum_{i=1}^{m}\left(x-1\right)+\sum_{i=1}^{r}x\right)}{x}, \end{array}$$

where *F*(*x*) represents the judgment function of determining the rule, *x* represents different processing samples, and *l* and *r* represent different selection rules.

In the above simulation analysis stage, the active participation of different types of college students in mental health services is simulated and analyzed by using the standard multidimensional intensity function value and fuzzy cluster analysis algorithm. The results are shown in Figure 3.

The star model based on fuzzy cluster analysis algorithm is adopted to realize the simulation analysis of the active participation of different types of college students in mental health services. The process of the results is shown in Figure 4.

On the other hand, according to the characteristics of the data group of college students' ideological and mental health support services, different methods can be used to modify, compensate, and classify them. The simulation analysis results are shown in Figure 5. The horizontal axis represents the data group of different types of college students' ideological and mental health support services, and the vertical axis represents the value of active participation.

It can be seen from Figures 3–5 that, for different types of college students' ideological and mental health support service enthusiasm data groups, the distance values of the standard function presented before and after are different, because for different types of college students' ideological and mental health support service data, the differences after star model analysis are easy to be distinguished. For example, in the same group, the disturbance of the results corresponding to the star discrete analysis model analysis method is the smallest.

## 4. Result Analysis and Discussion

### 4.1. Experiment on the Evaluation System of Active Participation of College Students' Mental Health Support Services Based on Star Discrete Analysis Model Based on Fuzzy Cluster Analysis Algorithm

After constructing the evaluation method of the active participation of college students' ideological and mental health support services based on star discrete analysis model based on fuzzy cluster analysis algorithm, it is necessary to analyze its effect on the real college students' ideological and mental health. Therefore, the system selects the ideological and mental health support service data of college students in a university as the original data, and the corresponding preliminary experimental results are shown in Figure 6. The horizontal axis represents the number of experiments, and the vertical axis represents the quantitative index of the active participation evaluation system.

As can be seen from Figure 6, under the analysis strategy of fuzzy clustering algorithm, with the increase of the number of experiments, the corresponding analysis results have different jumps, and the degree of change between the internal correlation star data group and the noncorrelation star data group is also significantly different. This is because, after adopting the star discrete analysis model based on fuzzy clustering analysis algorithm, its data analysis process has the law of discretization, so its internal relevance and universality also have a good coupling and normalization effect. After using Planck constant analysis, its error is effectively reduced from three dimensions, which greatly improves the accuracy of the analysis results.

### 4.2. Experimental Results and Analysis

In the process of analyzing the experimental results, the system selects the ideological and mental health support service data of college students in a university as the original data and sets different groups (experimental group and control group, in which the experimental group adopts star discrete analysis model and the control group adopts star continuous analysis model). The analysis results of the experimental data are shown in Figure 7. The horizontal axis represents the calculation and analysis times of different college students' ideological and mental health support service data, and the vertical axis represents the error analysis quantitative index of active participation.

Through the analysis of the data of college students' ideological and mental health support services in the results in Figure 7, it can be found that, under the star continuous analysis model of fuzzy cluster analysis algorithm, the data error degree of the experimental group and the control group will show strong disturbing characteristics with the internal correlation, and its internal data coupling error strategy will also have low-level discrete driving representation. Therefore, the accuracy of the result correlation is very high, while the deviation of the result correlation of the control group is very obvious [26]. Then we can know that, in the process of practical application, we need to combine the deviation of active participation of different types of college students' ideological and mental health support services to realize its quantitative evaluation and reliability disposal.

## 5. Conclusion

At present, there are some problems in the active participation of college students in ideological and mental health support services in China, such as low attention, low participation, and high data redundancy. Based on this, this paper studies the active participation of college students' ideological and mental health support service based on fuzzy cluster analysis algorithm. Compared with the disadvantages of the current mainstream discrete optimization analysis models on mental health (such as high-dimensional enterprise model, Dajiaweikang model, and short-range group control model), which need to set the known data gradient interval, this paper creatively adopts the fuzzy cluster analysis algorithm, based on the characteristics of different types of college students' ideological and mental health problems, combined with the improved star discrete analysis model, this paper constructs the active participatory evaluation strategy of college students' ideological and mental health support services. On this basis, the model can not only record and store the participatory data of ideological and mental health support for students of different grades, but also match and track different types of data based on special framework conditions, so as to achieve numerical normal analysis and directional matching for the data coupling mode of college students' ideological and mental health support services. On the other hand, the Planck constant factor is used to classify different types of ideological and psychological factor data, and combined with the idea of fuzzy clustering, the hierarchical analysis and quantitative calibration of different types of data groups are realized, so as to improve the reliability and authenticity of the active participation in college students' mental health support services. However, this study only studies the initiative of college students' ideological and mental health support services and does not analyze it from the perspective of passivity and relevance of different types of data groups. Therefore, more in-depth research can be carried out.

## Figures and Tables

**Figure 1:** The star discrete analysis model based on fuzzy clustering is used to support the data analysis process of service structure optimization.

**Figure 2:** Simulation analysis of active participation in support services with star discrete analysis model in quantitative evaluation.

**Figure 3:** The results of simulation analysis on the active participation of different types of college students' mental health services by using fuzzy clustering analysis algorithm.

**Figure 4:** Simulation results of the star model of fuzzy clustering analysis algorithm on the active participation of different types of college students in mental health services.

**Figure 5:** Simulation analysis results after correction, compensation, and classification by different methods.

**Figure 6:** Preliminary experimental results of active participatory evaluation of mental health support services for college students.

**Figure 7:** Functional analysis of experimental results.

## Data Availability

The figures used to support the findings of this study are included in the article.
